The article "Outcome of Extracorporeal Membrane Oxygenation Combined with Intraaortic Balloon Pump Hemodynamic Support during the Percutaneous Coronary Intervention Process for Patients with Cardiac Shock Complicating Acute Myocardial Infarction" was retracted in 2023. Reasons: signs of a paper mill; suspected computer-generated content; unreliable results or conclusions; lack of ethics approval or compliance.

# Outcome of Extracorporeal Membrane Oxygenation Combined with Intraaortic Balloon Pump Hemodynamic Support during the Percutaneous Coronary Intervention Process for Patients with Cardiac Shock Complicating Acute Myocardial Infarction

**DOI:** 10.1155/2022/1350673

**Published:** 2022-03-07

**Authors:** Minghua Luo, Jing Zhou, Chengjie Qiu, He Wang, Huaimin Guan, Yida Tang, Yushan Chen, Jinhong Xie, Yonghua Zong, Wenjie Dong, Shasha Shang, Gang Liu, Chunying Si

**Affiliations:** ^1^Department of Cardiology, The First Affiliated Hospital of Henan University of Chinese Medicine, Zhengzhou, Henan 450000, China; ^2^Department of Imaging, Henan Provincial Chest Hospital, Zhengzhou, Henan 450000, China; ^3^Department of Cardiology, Peking University Third Hospital, Beijing 100109, China

## Abstract

We evaluate the effect of extracorporeal membrane oxygenation combined with intraaortic balloon pump mechanical circulatory support for patients with cardiogenic shock complicating acute myocardial infarction during the PCI process. Extracorporeal membrane oxygenation combined with intraaortic balloon pump hemodynamic support during the percutaneous coronary intervention process for patients with cardiac shock complicating acute myocardial infarction might play a complementary role. Yet, evidence of application of both devices at the same time remains unclear. Patients with cardiogenic shock complicating myocardial infarction who underwent PCI in our hospital from January 2015 to January 2018 were screened. Those who were under hemodynamic support of extracorporeal membrane oxygenation combined with intraaortic balloon pump were enrolled as the ECMO&IABP group, and the patients only under support of intraaortic balloon pump were enrolled as the IABP group. The differences of clinical prognosis between the two groups were compared. A total of 39 patients were enrolled into the study: 10 were in the ECMO&IABP group and 29 in the IABP group. Compared with the IABP group, more patients were complicated with old myocardial infarction (5/10 vs. 2/29, *p*=0.002), more patients were diagnosed as non-ST elevated myocardial infarction (8/10 vs. 11/29, *p*=0.002) and left ventricular ejecting fraction was lower (41.1 ± 9.86 vs. 48.55 ± 8.86, *p*=0.03) in the ECMO&IABP group. Mechanical complications were higher in the ECMO&IABP group (5/10 vs. 5/29, *p*=0.048), The survive rate in the ECMO&IABP group is higher than that in the IABP group (90.00% vs. 47.83%, *p*=0.042) at one-year follow-up. Compared with only IABP, ECMO combined with IABP hemodynamic support during the PCI process for patients with cardiogenic shock complicating acute myocardial infarction enjoys better mortality outcome.

The article "Outcome of Extracorporeal Membrane Oxygenation Combined with Intraaortic Balloon Pump Hemodynamic Support during the Percutaneous Coronary Intervention Process for Patients with Cardiac Shock Complicating Acute Myocardial Infarction" was retracted in 2023. Reasons: signs of a paper mill; suspected computer-generated content; unreliable results or conclusions; lack of ethics approval or compliance.

## 1. Introduction

Patients with acute myocardial infarction (AMI) complicated with cardiogenic shock (CS) suffer very high rate of mortality [1]. Myocardial ischemia induces profound depression of myocardial contractility, which initiates a vicious spiral of reduced cardiac index and low blood pressure which further promote coronary ischemia. The reduction in cardiac index causes severe tissue hypoperfusion and may finally lead to MODS and even death if the vicious circle is not successfully interrupted by adequate treatment. Revascularization is of vital to reduce death and improve prognosis [2, 3]. However, such patients are already in or on the verge of very critical heart failure and circulatory collapse, and revascularization will be at great risk. Thus, mechanical circulatory support is critically needed.

We assume that ECMO with IABP support during the PCI procedure might change the dismal prognosis of patients with CS complicating AMI. At present, data about this are limited. In this retrospective case study, we try to explore the clinical outcome of patients with CS complicating AMI who were under the support dual-device of ECMO and IABP during the PCI process.

The rest of the study is structured as follows.  Section 2 provides materials and methods of this research.  Section 3 presents the results of this research. Data analysis is described in Section 4. Last, we conclude this research and point out some potential future research directions in Section 5.

## 2. Materials and Methods

### 2.1. Patients

Patients with AMI complicated with CS who underwent primary PCI in our hospital from January 2015 to January 2018 were screened. Those who were under hemodynamic support of ECMO combined with IABP were enrolled into the ECMO&IABP group, and the patients who were only under support of IABP were enrolled into the IABP group. The demographic information, hemodynamic data, and coronary angiography were summarized. Then, the differences of clinical prognosis between the two groups were compared. This investigation was in accordance with the Declaration of Helsinki.

### 2.2. Definitions

Diagnosis of CS was according to the following established criteria [4]: systolic blood pressure<90 mmHg for 30 min or vasopressors required to achieve a blood pressure ≥90 mmHg, pulmonary congestion or elevated left ventricular filling pressures, and signs of impaired organ perfusion with at least one of the following criteria: altered mental status; cold, clammy skin; oliguria; and increased serum-lactate.

### 2.3. IABP and ECMO Insertion and Weaning

Patients were well prepared with mechanical support of IABP (CS100, Intelligent Counterpulsation, MAQUET) or VA-ECMO (CBIQ91R6 kit, Medtronic Minimax PlusOxygenator, Medtronic Inc, Minneapolis, USA) with IABP immediately before PCI procedure. Before femoral tube insertion, using the preembedded suture technique, two Perclose ProGlide suture-mediated closure systems (ProGlide, Abbott) were intercrossly sutured. The activated clotting time (ACT) was adjusted to about 180–220 seconds with intravenous heparin. ECMO flow was downregulated according to the daily monitoring results of cardiac function changes and arterial blood gas. ECMO support was weaned when the flow was less than 1.5 L/min, and hemodynamics was stable with little or no vasoactive treatment. Successful mechanical support withdrawal is defined as the survival time is more than 48 hours after the withdrawal.

The article "Outcome of Extracorporeal Membrane Oxygenation Combined with Intraaortic Balloon Pump Hemodynamic Support during the Percutaneous Coronary Intervention Process for Patients with Cardiac Shock Complicating Acute Myocardial Infarction" was retracted in 2023. Reasons: signs of a paper mill; suspected computer-generated content; unreliable results or conclusions; lack of ethics approval or compliance.

### 2.4. Observational Parameters

The general data of the two groups were compared, including gender, age, BMI, coronary risk factors, eGFR, GRACE score, Killip grade, peak value of myocardial injury markers, and so on. The special data were compared, including SYNTAX score, target vessel, IABP using duration, ECMO using duration, successful rate of mechanical weaning, and in-hospital mortality. The one-year follow-up survival rate between the two groups was compared.

### 2.5. Statistical Analysis

Data are summarized as number (percentages) for categorical variables. Continuous variables are expressed as median (interquartile range). Qualitative data are compared using the *x*^2^ or Fisher exact tests, while quantitative data are compared using the Mann–Whitney *U* test. The survival rate is described by Kaplan–Meier curve, and the survival curve is compared by the log rank test. All analyses are performed by SPSS Statistics (ver. 22; IBM Co., NY, USA). Statistical significance is established at *p* < 0.05 (two-tailed).

## 3. Experimental Results

### 3.1. Baseline, Procedural Characteristics, and In-Hospital Outcomes

A total of 29 patients (median age 66 (48–84) years) and 10 patients (median age 64.5 (30–83) years) were included in the IABP and ECMO&IABP groups, respectively. Comparison of baseline and procedural characteristics of patients as well as in-hospital outcomes between the two groups is given in Table 1. In the ECMO&IABP group, more patients were complicated with previous myocardial infarction (50% vs. 6.90%, *p*=0.002) than that in the IABP group. More patients in the ECMO&IABP group were diagnosed as NSTEMI (80% vs. 37.93%, *p*=0.02), while less STEMI (20% vs. 62.07%, *p*=0.02) in comparison with the IABP group. The rate of multivessel disease and the SYNTAX score in the ECMO&IABP group was higher than that in the IABP group (8/10 vs. 11/29, *p*=0.02) (31.80 ± 12.99 vs. 25.74 ± 5.75, *p*=0.049). The in-hospital outcomes showed longer duration of IABP application (65.90 ± 56.45 vs. 31.62 ± 29.76, *p*=0.019) and longer stay in hospital of patients in the ECMO&IABP group than that in the IABP group (25.00 ± 17.51 vs. 14.17 ± 12.32, *p*=0.046). Mechanical complications were higher in the ECMO&IABP group.

The article "Outcome of Extracorporeal Membrane Oxygenation Combined with Intraaortic Balloon Pump Hemodynamic Support during the Percutaneous Coronary Intervention Process for Patients with Cardiac Shock Complicating Acute Myocardial Infarction" was retracted in 2023. Reasons: signs of a paper mill; suspected computer-generated content; unreliable results or conclusions; lack of ethics approval or compliance.

### 3.2. Survival Outcomes

The survive rate of patients in the ECMO&IABP group was higher than that in the IABP group (90.00% vs. 47.83%, *p*=0.042 at one-year follow-up, as shown in Figure 1. There was no death in the ECMO&IABP group during 12 months follow-up; whereas, in the IABP group, two patients died at 1 month and 3 patients die at 12 months, as given in Table 2. Cause of death analysis shows that 1 patient in ECMO&IABP died of hemorrhagic shock when in hospital. In the IABP group, 3 died of cardiac arrest, 1 cardiac rupture, and 2 pump failure in hospital; 1 sudden death and 1 cardiac arrest at 1 month follow-up; 2 sudden death and 1 stoke at 12 months follow-up.  Table 3 presents number and cause of death during 12 months follow-up.

### 3.3. Complications

The rate of complications in the ECMO&IABP group is higher than that in the IABP group (5/10 vs. 5/29, *p*=0.048). In the ECMO&IABP group, there was one patient complicated with lower limb ischemia, one with pulmonary hemorrhage, one with subcutaneous hemorrhage, and one with upper gastrointestinal hemorrhage; five patients were transfused. While in the IABP group, one patient was complicated with hematoma at the femoral puncture site, one with major gastrointestinal bleeding, one with acute liver injury, and one with pulmonary infection.

## 4. Experimental Results and Discussion

According to our analysis, compared with only IABP hemodynamic support, ECMO combined with IABP support reduces the mortality of patients with cardiac shock (CS) complicating AMI during the PCI process, which provides evidence for reconsideration of such mechanical circulatory support (MCS) for patients under similar conditions.

Standard therapy for cardiac shock (CS) consists of primarily volume management as well as inotropic agents and vasopressors enhancing cardiac output and the vascular tone. MCS is an alternative to increase blood flow avoiding the possible cardiotoxicity of inotropes and vasopressors, and it seems to be the only way to achieve hemodynamic stability in patients with CS. However, evidence on the role of active MCS in patients with CS compared with standard therapy is limited [1]. IABP has been the most widely used MCS for nearly 5 decades, which is conventionally considered to improve the diastolic pressure and lower the end systolic pressure without affecting the mean blood pressure. However, IABP does not actively provide cardiac support and fails to function in case of cardiac arrest or ventricular fibrillation. Moreover, IABP depends on a certain amount of residual left ventricular function. As a result, it is difficult to provide stable and effective circulatory support for cardiogenic shock patients. Nowadays, its effect is still in controversial. A meta-analysis shows that IABP is associated with significantly improved in-hospital mortality when used in AMI with CS, but it is also associated with a significant increase in the risk of moderate and major bleeding [5]. The IABP-SHOCK II trial shows that IABP does not reduce 30-day and 12-month all-cause mortality [6]. Therefore, guidelines discourage the routine use of IABP as a first-line treatment in CS patients and emphasizes the application should be restricted to those patients with refractory shock [7].

The article "Outcome of Extracorporeal Membrane Oxygenation Combined with Intraaortic Balloon Pump Hemodynamic Support during the Percutaneous Coronary Intervention Process for Patients with Cardiac Shock Complicating Acute Myocardial Infarction" was retracted in 2023. Reasons: signs of a paper mill; suspected computer-generated content; unreliable results or conclusions; lack of ethics approval or compliance.

Extracorporeal membrane oxygenation (ECMO) provides continuous perfusion blood with sufficient oxygen even under the condition of the very low cardiac output, such as severe pump failure, malignant arrhythmias, and cardiac arrest. However, ECMO has some defects. First, the advection perfusion does not increase the diastolic pressure of the heart, on which the coronary perfusion mainly depends on. Second, ECMO increases afterload which could lead to inadequate LV unloading and make it worse for the impaired heart function. However, IABP increases diastolic blood pressure which benefits coronary artery perfusion; it also has the potential of reducing systolic blood pressure, which means reduction of left ventricular afterload and myocardial oxygen consumption, thereafter contributing to recovery of cardiac function.

As analyzed above, ECMO combined with IABP provides both complementary hemodynamic support and myocardial protection which might play a complementary role during the process of PCI. Yet, evidence of application of both devices at the same time still remains unclear. One observational analysis shows that the routine insertion of concomitant IABP with ECMO is not supported because the concomitant use of IABP with ECMO does not appear to be associated with a dramatic change in survival outcomes [8]. However, physiological studies demonstrated left ventricular afterload decreasing during ECMO assistance combined with the IABP, and associating IABP with VA-ECMO was independently related to a lower frequency of hydrostatic pulmonary edema and more days off mechanical ventilation [9]. Another study showed the use of IABP combined with ECLS achieved an early effective hemodynamic support; it was an independent protective factor for patients with CS complicating AMI [10]. A lately meta-analysis shows that in patients with AMI, use of IABP with VA-ECMO is associated with 18.5% lower mortality in comparison to patients on VA-ECMO alone [11]. Recently, the utility of device use in combination for patients with severe CS has been recognized; in most CS cases, any MCS device alone may be insufficient to correct the hemodynamic abnormality following AMI [12]. The dual‐device approach allows for a stepwise deescalation of support as the patients recover, so it is very important to keep close hemodynamic monitoring after application of one device. Our study indicates the positive effect of ECMO combined IABP support for patients with CS following AMI, which benefits lower 12 months mortality compared with only under support of IABP.

The article "Outcome of Extracorporeal Membrane Oxygenation Combined with Intraaortic Balloon Pump Hemodynamic Support during the Percutaneous Coronary Intervention Process for Patients with Cardiac Shock Complicating Acute Myocardial Infarction" was retracted in 2023. Reasons: signs of a paper mill; suspected computer-generated content; unreliable results or conclusions; lack of ethics approval or compliance.

Revascularization has dramatically improved outcome and reduced in-hospital mortality of CS patients following AMI from 70–80% to 40–50% [4]. The landmark SHOCK trial demonstrated a mid to long-term survival advantage for revascularization versus medical stabilization, and the increase in PCI for this condition has resulted in a significant decline in mortality [13, 14]. 2018 ESC/EACTS guidelines on myocardial revascularization recommend that PCI of the culprit lesion is indicated for patients with cardiogenic shock due to STEMI or NSTE-ACS, independent of time delay of symptom onset, if coronary anatomy is amenable to PCI [15–17]. All the patients enrolled in our study were under revascularization. Both groups show high SYNTAX score, and more patients in the ECMO&IABP group show multivessel coronary disease [18]. We assume that the existence of recoverable myocardium should be a great concern on whether MCS should be applied or not. The less myocardium infarcts, the more likely the heart function recovers.

Complications brought by devices must be paid as much attention as possible to avoid, so that the benefit could outweigh complications. Sometimes, those complications are very fatal [19–21]. Actually, in our study, one patient in the ECMO&IABP group died of bleeding which was caused by insertion of the ECMO tube. The better outcome requires a multidisciplinary approach to prevent complications especially caused by the device itself and to limit organ injury before and during support. Consideration must be put to identify appropriate candidates for VA-ECMO support to avoid unnecessary use. The advantages and disadvantages as well as safety and efficacy of different MCS devices should be well acknowledged.

## 5. Conclusion

This study is a retrospective analysis in which the cohorts are not randomized and the number of cases is small; thus, the statistical bias is unavoidable. In the study, most of the patients in the ECMO&IABP group were NSTEMI, indicating that when we applied ECMO combined with IABP, we are prone to choose the patients with less myocardial infarction and more myocardial stunning, and the cardiac functions of these patients were more recoverable. Compared with only IABP, ECMO combined with IABP hemodynamic support during the PCI process reduces 12 months mortality of patients with CS complicating AMI.

The article "Outcome of Extracorporeal Membrane Oxygenation Combined with Intraaortic Balloon Pump Hemodynamic Support during the Percutaneous Coronary Intervention Process for Patients with Cardiac Shock Complicating Acute Myocardial Infarction" was retracted in 2023. Reasons: signs of a paper mill; suspected computer-generated content; unreliable results or conclusions; lack of ethics approval or compliance.

## Figures and Tables

**Figure 1:** The survival curve of patients within two groups. ECMO, extracorporeal membrane oxygenation; IABP, intraaortic balloon pump.

**Table 1:** Baseline, procedural characteristics, and in-hospital outcomes of the IABP and ECMO&IABP groups.

Variables	IABP group (*n* = 29)	ECMO&IABP group (*n* = 10)	*P* value
Baseline characteristics			
Clinical characteristics			
Age (years)	66 (48–84)	64.5 (30–83)	0.45
Female sex	10	1	0.14
Body mass index (kg/m^2^)	24.77 ± 2.22	25.25 ± 3.54	0.63
Hypertension	21	7	0.88
Diabetes mellitus	6	4	0.23
Dyslipidaemia	2	1	0.75
Current smoker	11	6	0.22
Previous myocardial infarction	2	5	0.002^*∗*^
COPD	2	1	0.75
Previous stroke/TIA	9	3	0.95

Presentation			
STEMI	18	2	0.02^*∗*^
NSTEMI	11	8	0.02^*∗*^
Electrical cardioversion	8	2	0.64

Killip classification			
III	13	7	0.17
IV	16	3	0.17
Heart rate (bpm)	83.97 ± 19.22	85.6 ± 23.71	0.83
Systolic BP (mmHg)	89.52 ± 17.89	85.20 ± 9.22	0.47

Blood tests			
P-CK	2954.95 ± 3134.36	886.70 ± 1210.37	0.005^*∗*^
P-CKM B	245.21 ± 250.34	38.67 ± 29.65	0.01^*∗*^
P-cTnt	40.50 ± 42.09	36.58 ± 83.30	0.86
eGFR	77.40 ± 29.59	82.19 ± 18.36	0.64

Procedure characteristics			
Infarct-related coronary artery			
Left anterior descending	24	10	0.16
Left circumflex	8	6	0.065
Right	8	6	0.065
Left main	4	4	0.077
SYNTAX score	25.74 ± 5.75	31.80 ± 12.99	0.049^*∗*^
Multivessel disease	11	8	0.02^*∗*^

In-hospital outcomes			
Duration of ECMO (h)	—	30.20 ± 28.03	—
Duration of IABP	31.62 ± 29.76	65.90 ± 56.45	0.019^*∗*^
Successful mechanical weaning	21	9	0.21
Left ventricular EF (%)	48.55 ± 8.86	41.1 ± 9.86	0.03^*∗*^
Left ventricular EF <35%	3	4	0.035^*∗*^
Length of stay (days)	14.17 ± 12.32	25.00 ± 17.51	0.046^*∗*^
Mechanical complications	5	5	0.048^*∗*^
Cardiovascular mortality	10	1	0.138

^*∗*^ *P* < 0.05. ECMO, extracorporeal membrane oxygenation; IABP, intraaortic balloon pump; COPD, obstructive pulmonary disease; TIA, transient ischemic attack; STEMI, ST-segment elevation myocardial infarction; NSTEMI, non-ST-segment elevation myocardial infarction.

**Table 2:** Survival rate of the two groups during 12 months follow-up.

	Discharge	1 m	2 m	6 m	12 m
IABP group (*n* = 29)	19 (69.57%)	18 (60.87%)	18 (60.87%)	18 (60.87%)	17 (47.83%)
ECMO&IABP group (*n* = 10)	9 (90%)	9 (90%)	9 (90%)	9 (90%)	9 (90%)

The article "Outcome of Extracorporeal Membrane Oxygenation Combined with Intraaortic Balloon Pump Hemodynamic Support during the Percutaneous Coronary Intervention Process for Patients with Cardiac Shock Complicating Acute Myocardial Infarction" was retracted in 2023. Reasons: signs of a paper mill; suspected computer-generated content; unreliable results or conclusions; lack of ethics approval or compliance.

**Table 3:** Number and cause of death during 12 months follow-up.

	Inhospital	1 m	2 m	6 m	12 m
IABP group (*n* = 29)	Cardiac arrest (3)				
	Cardiac rupture (1)	Sudden death (1)	0	0	Sudden death (2)
	Pump failure (2)	Cardiac arrest (1)			stroke (1)
	Stroke (1)				
ECMO&IABP group (*n* = 10)	Hemorrhagic shock (1)	0	0	0	0

## Data Availability

The simulation experiment data used to support the findings of this study are available from the corresponding author upon request.
